# Evaluation of Oncogene NUP37 as a Potential Novel Biomarker in Breast Cancer

**DOI:** 10.3389/fonc.2021.669655

**Published:** 2021-07-27

**Authors:** Kangdi Li, Ting Liu

**Affiliations:** ^1^GI Cancer Research Institute, Tongji Hospital, Huazhong University of Science and Technology, Wuhan, China; ^2^The Central Hospital of Wuhan, Tongji Medical College, Huazhong University of Science and Technology, Wuhan, China

**Keywords:** breast cancer, NUP37, prognostic marker, therapeutic target, cell growth, cell migration

## Abstract

**Purpose:**

There is an urgent need to identify oncogenes that may be beneficial to diagnose and develop target therapy for breast cancer.

**Methods:**

Based on the GEO database, DECenter was used to screen the differentially overexpressed genes in breast cancer samples. Search Tool for the Retrieval of Interacting Genes and Cytoscape were performed to construct the PPI network to predict the hub gene. Functional and pathway enrichment were performed based on GO analysis. GEO2R, Oncomine, human tissue microarray staining, and western blot were applied to confirm the expression of NUP37. The association between NUP37 expression and prognosis in patients with breast cancer were assessed using the Kaplan–Meier plotter online tool and OncoLnc. siRNAs were used to knock down NUP37 and evaluate proliferation, migration, and stemness in breast cancer cells.

**Results:**

We found that 138 genes were differentially upregulated in breast cancer samples, mainly comprising components of the nucleus and involved in the cell cycle process. NUP37 was identified as a hub gene that is upregulated in breast cancer patients related to a significantly worse survival rate. Furthermore, we confirmed that the downregulation of NUP37 in breast cancer cells results in the inhibition of cell growth, migration, and stemness.

**Conclusions:**

High expression of NUP37 in breast cancer patients is associated with a poorer prognosis and promotion of cell growth, migration, and stemness. The multiple bioinformatics and experimental analysis help provide a comprehensive understanding of the roles of NUP37 as a potential marker for diagnosis and prognosis and as a novel therapeutic target in breast cancer.

## Introduction

Breast cancer (BRCA) is the most frequently diagnosed cancer in women and is one of the most common causes of cancer-related mortality worldwide (1). Although great advances have been made in past decades, there remains an urgent need to identify new oncogenes and explore their molecular mechanisms in the development and progression of BRCA. It is expected that these genes may be beneficial to diagnosis and the discovery of effective therapeutic targets in BRCA treatment (2).

Recently, the application of developed gene microarrays and bioinformatics analysis have been considered valid approaches for cancer research (3–6). Studies based on public data such as high-throughput data from the NCBI Gene Expression Omnibus (GEO) and The Cancer Genome Atlas (TCGA) have been combined with statistical analytical tools (7, 8). Broadly screening differentially expressed genes and evaluating prognostic values of target genes made it possible to predict the benefit biomarkers of cancers (9–11).

We aimed to apply the computational bioinformatics methods to explore the target genes and identify key genes with a prognostic value for the survival of BRCA patients. First, we used the statistical software DECenter based on microarray datasets obtained from GEO datasets GSE73613 and GSE41445 in the Gene Expression Omnibus (GEO) database to screen differentially expressed genes (DEGs) between BRCA and normal samples. Next, we predicted the hub genes of the DEGs based on the protein-protein interaction (PPI) network using Search Tool for the Retrieval of Interacting Genes (STRING) and Cytoscape and function and component enrichment analysis based on Gene Ontology (GO). GEO2R and Oncomine were applied to verify the overexpression level of the target gene NUP37 in BRCA compared with normal samples. Subsequently, the association between NUP37 and recurrence-free survival (RFS), distant metastasis-free survival (DMFS), and overall survival (OS) in BRCA patients were assessed using the Kaplan–Meier plotter online tool and Oncolnc (**Figure 1A**). Furthermore, we analyzed the proteins that directly interact with NUP37 and genes co-expressed with NUP37 by STRING and Multi Experiment Matrix (MEM), respectively. Function analysis of the co-expressed genes was performed using Metascape for annotation. Finally, we identified PSMG1, one of the genes co-expressed with NUP37, as having a highly positive relationship with NUP37 in The Cancer Genome Atlas- Breast Cancer (TCGA-BRCA) database using Xena.

Nuclear pore complexes (NPCs) are supramolecular structures that fuse the inner and outer nuclear membranes to form channels embedded in the nuclear envelope. NPCs are composed of multiple copies of about 30 different proteins termed nucleoporins (Nups) that serve as the primary transport gates for nucleocytoplasmic molecular exchange (12). Besides the main role of NPCs in regulating molecular trafficking between nuclear and cytoplasm, NPCs and their components also play important transport-independent roles, including gene expression regulation, chromatin organization, DNA repair, RNA processing and quality control, and cell cycle control (13). As the largest subunit of the NPC, the Nup107-160 subcomplex (Y-complex) is a core building block of the NPC and multifunctional. It mediates mRNA export in interphase, and has roles in kinetochore function, and is critical for spindle assembly and postmitotic nuclear pore assembly (14). NUP37 (Nucleoporin 37 kDa), the identified target gene in this research, coded protein Nup37, is one of the nine components of the Nup107-160 subcomplex; it is specific to higher eukaryotes and lacking in plant (15). Nup37 binds to the Nup120 protein, which is a subunit that forms one of the two short arms of the Y-complex, to potentially stabilize the relative orientation of its two domains (16). It has been reported that Nup37 with all constituents of Nup107-160 complex, targeted to kinetochores from prophase to anaphase of mitosis (17). The role of Nup37 has rarely been reported in cancer cells and has never been studied in BRCA previously. Luo et al. demonstrated NUP37 as a positive regulator of YAP/TEAD signaling in promoting the progression of hepatocellular carcinoma (18), and the Chen group also found liver cancer cell proliferation could be inhibited *via* destabilizing NUP37 (19). In non-small cell lung cancer cells, the silence of NUP37 results in inhibition of cell proliferation, G1 phase cell cycle arrest, and apoptosis (20). Interestingly, we found a high expression of NUP37 in BRCA associated with a poor prognosis. Additionally, we assessed the gene PSMG1(Proteasome assembly chaperone 1), alternatively named C21LRP, DSCR2, which encodes proteasome (prosome, macropain) assembly chaperone 1 and promotes assembly of the core catalytic 20S proteasome as part of a heterodimer with PSMG2 (21), was highly co-expressed with NUP37 in BRCA samples. This bioinformatics analysis provided evidence to show that NUP37 may act as a biomarker for the diagnosis and outcomes in BRCA, and PSMG1 might be involved in the oncogenic pathway of NUP37 in BRCA.

Breast cancer cells are known to have properties such as high proliferation rate, increased cell migration, and capacity of epithelial-mesenchymal transition (EMT) and tumor-initiating cell stemness (22). In order to confirm the bioinformatics analysis, here, cell culture studies have been used to investigate the effects of NUP37 on the properties of breast cancer cells by siNUP37. The capacity of EMT can be evaluated by the expression of EMT-related markers. Reverse EMT, which resulted in a decrease in the levels of mesenchymal markers such as Vimentin and N-cadherin and an increase in the levels of epithelial markers such as Occludin and E-cadherin in the cells (23). The cancer cell stemness can be assessed by mammosphere forming efficiency and the cancer stem cells surface marker CD44^+^CD24^-/low^ subpopulation (24). Our study showed that siNUP37 inhibited cell proliferation and migration, downregulated EMT properties, and attenuated stemness of breast cancer cells. We need further experimental evaluation for the potential use of NUP37 and its underlying mechanism in the diagnosis and treatment of BRCA.

## Materials and Methods

### DEGs Screening

BRCA-associated gene expression profiles (GSE73613 and GSE41445) were downloaded from Gene Expression Omnibus (GEO, http://www.ncbi.nlm.nih.gov/geo/) database in the National Center for Biotechnology Information (NCBI). DECenter based on R language was applied to significance analysis of DEGs between BRCA samples and normal samples. P < 0.05 and logFC > 2 was considered statistically significant. GSE73613 included expression data from two normal breast tissues and two invasive primary breast carcinoma tissues. GSE41445 included expression data from 21 cell lines (18 cancer and 3 non-tumorigenic).

### Protein–Protein Interaction (PPI) Network Analysis

PPI information was acquired from the Search Tool for the Retrieval of Interacting Genes (STRING) online database (http://www.stringdb.org/), which provides information for experimental and predicted interactions. Specifically, we firstly type a list of DEGs or a single protein name in the search box and choose the corresponding species, then the String website will query the database and return the matching network to construct a network for protein interactions and generate a string file in tsv format, which can help us identify the key genes and the important gene involved in BRCA development from interaction level. Next, we exported string interactions in tsv format in the exports interface and imported this tsv file to Cytoscape software to visualize the construction of the PPI network and perform an interaction score calculation. Genes with the top 10 degrees were displayed as bigger circles.

### Gene Expression Analysis

GEO2R (https://www.ncbi.nlm.nih.gov/geo/geo2r/) is a web tool that is applied to screen genes by comparing two groups of samples. Firstly, enter a series accession number in the box. Then, click “Define groups” and enter names for the BRCA and normal groups of samples to compare. After samples have been assigned to groups, click “Profile graph” and enter the gene ID of NUP37 to get the expression value, then use Graphpad to generate the graph.

NUP37 gene expression in BRCA specimens and normal tissues is also available through Oncomine. (Compendia Biosciences, www.oncomine.org), the cut-off p-value and fold change were defined as 0.01 and 2, respectively.

### Human Tissue Microarray Immunohistochemical Staining

Human tissue specimens (HBreD090CS01) were purchased from Shanghai Outdo Biotech CO. The primary antibody anti-Nup37 (Abcam, ab220675) was diluted at 1:20. The standard IHC procedure was performed according to the manufacturer’s instructions (Dako). The tissue samples were examined by two pathologists, and the Nup37 expression level of each tissue sample was scored according to its staining intensity (0, none; 1, weak; 2, moderate; 3, strong) and the percentage of stained cells (0, 0%; 1, 1-24%; 2, 25-49%; 3, 50-74%; 4, 75-100%). Then, the final value between 0 and 12 was calculated by multiplying the staining intensity and the percentage of stained cells.

### Gene Annotation and Analysis

The biological significance of DEGs was explored by GO term enrichment analysis to illuminate the biological process, cellular component, and molecular function based on using STRING. Metascape also provides a web portal for gene annotation and analysis resources that help to make sense of multiple gene lists.

### Survival Analysis

The Kaplan-Meier plotter (KM plotter) online web tool predicts the effect of genes on survival (http://kmplot.com/analysis/index.php?p=background). By entering NUP37 to the blanks on the website and checking the ER status option, patients were divided into two groups according to the expression level of the gene, and we statistically analyzed the RFS and DMFS. The hazard ratio (HR) with 95% confidence intervals and logrank P values were calculated and showed. Besides, using OncoLnc, another online web tool, submitting NUP37 and clicking BRCA to link the TCGA survival data, we compares the OS by choosing bottom third *versus* top third of patients sorted by NUP37 expression.

### Identification of Co-Expressed Genes

As a system biology method, gene co-expression network analysis was performed by MEM (https://biit.cs.ut.ee/mem/), a web-based multi experiment gene expression query and visualization tool that gathers several hundreds of publicly available gene expression data sets from ArrayExpress database based on different tissues, diseases, and conditions. We entered the NUP37 gene ID into the text field and selected H.sapiens, chose the A-AFFY-44 collection, put the data list as query in 100 pop-ups, and then submitted; the co- expressed genes were sequenced by their P value. Finally, we applied Xena online tool (http://xena.ucsc.edu/) to further validate the co-expression relationship with NUP37 and PSMG1. Afterwards, we selected Breast Cancer (BRCA- 1,247 samples), added NUP37 and PSMG1, and selected the assay type based on gene expression. Column A represents the sample, Column B is sorted according to NUP37 expression, and Column C is sorted according to PSMG1. Finally, generate the NUP37- PSMG1 gene expression line with Pearson’s rho and Spearman’s rank rho value.

### Cell Lines and Cell Culture

The breast cancer cell lines MCF10A, MDA-MB-231, MCF7, BT-549, ZR-75-30, and T47D were cultured at 37°C in a humidified atmosphere of 95% air and 5% CO2 in a complete 1640 RPMI medium (Gibco BRL, Grand Island, NY, USA) that was supplemented with 10% FBS (HyClone), 1% penicillin, and 1% streptomycin.

### Western Blot Analysis

Cells were harvested and lysed in 1% SDS on ice and then were heated at 98°C for 20 min. We collected the supernatant after the lysates were clarified by centrifugation at 12000g for 15 min, and the protein concentration was determined by the Pierce BCA Protein Assay Kit (Thermo Fisher Scientific, Waltham, MA, USA). Equal amounts of protein from each sample were separated on SDS-PAGE gels and transferred to PVDF membranes (Millipore, Billerica, MA, USA) and blocked for 1 h with 5% non-fat milk (Bio-Rad, Hercules, CA, USA) in Tris-buffered saline with 0.1% Tween 20 (TBST) at room temperature. Membranes were incubated with specific primary antibodies overnight at 4°C. The membranes were then washed with TBST three times (10 min every time) and incubated for 1 h with HRP-conjugated secondary antibodies at room temperature. After being washed with TBST, signals were visualized in the samples by chemiluminescent detection using an HRP substrate (Millipore). GAPDH was applied to ensure equal protein loading.

### Cell Proliferation Detection

Cell proliferation was measured by counting the total number of viable cells observed by the trypan blue dye exclusion assay, and 1 × 10^3^ BT549 and ZR-75-30 cells were plated on 96-well plates and transfected with siRNAs for the times indicated. Cells without trypan blue staining were then counted using a haemocytometer.

### Cell Migration Assay

For the wound-healing assays, 2.5 ×10^5^ cells were plated in a 12-well plate then a scratch was created by scraping the cells with a 200-μl pipette tip. The floating cells were gently rinsed away with PBS, and fresh medium was added. The width of the scratch was recorded at 0 h and 24h or 36 h. The migration rate was calculated by comparing the scratch area of the experimental group with the control group, and the migration rate of the control group has been set to 100%.

For the transwell migration assays, 5 × 10^4^ cells were suspended in 500 μL of FBS-free DMEM and plated in the upper chamber of transwell inserts (353097, Falcon). Then, 600 μL of completed medium was added to 24-well plates. After 24h and 36 h of incubation, the cells were fixed and stained according to the manufacturer’s protocols. Three randomly selected fields were photographed.

### FACS Analysis and Mammosphere Assay

For CD44^high^/CD24^low^ cell detection, cells were washed with PBS and stained with antibodies against CD24 (5554728, BD, NY, USA) and CD44 (555478, BD) for 15 min. The stained cells were then assessed by flow cytometry.

For mammosphere assay, 3× 10^3^ cells were suspended in culture medium mixed with EGF、FGF and B-27™ Supplement (12587010, Gbico) and plated in ultra-low attachment 6-well plates (3471, Coring). After 7 days of incubation, the mammospheres were photographed and counted.

## Results

### DEGs Screening, Enrichment Analysis, and PPI Network Identification in Breast Cancer

Firstly, by using statistical software DECenter, we identified a total of 138 up-regulated DEGs from both GSE73613 and GSE41445 datasets in the GEO database (**Figure 1B**). By using STRING and Cytoscape to construct the protein-protein interaction (PPI) network of DEGs, we focused on NUP37, one of the top 10 core genes located in the key nodes with a high degree (**Figure 1C**). According to the GO analysis which applied to reveal biological functions of genes, all up-regulated DEGs were classified into cellular components and biological processes. The results showed that the 138 up-regulated DEGs were primarily enriched in the cellular component of the nuclear part and in the biological process of the cell cycle (**Tables 1** and **2**). In consist of component and function enrichment, the hub gene NUP37 is a component of the nuclear pore complex, which may be involved in cell division (17). Thus, we suspect NUP37 may have a positive effect on tumorigenesis.

**Figure 1:** Gene screening and identification of the hub gene. **(A)** Illustrates the screening process of key gene in a simplified sequence flow diagram. **(B)** Identification of up-regulated DEGs in BRCA compared with normal control samples from GEO datasets (GSE73613, GSE41445). **(C)** PPI networks map of upregulated DEGs. The top 10 node genes with higher degrees are labeled in yellow, and the degree of the top 10 node genes are listed.

**Table 1:** Component annotation of 138 differentially expressed genes.

#PathwayID	Pathwaydescription	Observed gene count	False discovery rate
GO.0044428	nuclear part	51	7.66E-07
GO.0005634	nucleus	71	2.33E-06
GO.0031981	nuclear lumen	47	2.33E-06
GO.0044446	intracellular organelle part	75	4.05E-06
GO.0005654	nucleoplasm	41	6.89E-06
GO.0043231	intracellular membrane-bounded organelle	90	7.05E-06
GO.0070013	intracellular organelle lumen	50	7.81E-06
GO.0044424	intracellular part	99	3.77E-05
GO.0043227	membrane-bounded organelle	93	6.23E-05
GO.0005622	intracellular	100	6.24E-05

**Table 2:** Process annotation of 138 differentially expressed genes.

#Pathway ID	Pathway description	Observed gene count	False discovery rate
**GO.0000278**	mitotic cell cycle	21	0.000174
**GO.0007049**	cell cycle	26	0.000218
**GO.0022402**	cell cycle process	22	0.00055
**GO.1903047**	mitotic cell cycle process	18	0.00102
**GO.0044260**	cellular macromolecule metabolic process	64	0.00138
**GO.0007093**	mitotic cell cycle checkpoint	9	0.00192
**GO.0000075**	cell cycle checkpoint	10	0.00203
**GO.0008152**	metabolic process	79	0.00272
**GO.1903320**	regulation of protein modification by small protein conjugation or removal	10	0.00589
**GO.0043170**	macromolecule metabolic process	65	0.0062

### The Expression of NUP37 Is Upregulated in Breast Cancer

To verify the expression of NUP37 in BRCA, we analyzed NUP37 between normal and BRCA samples from GSE73613, GSE41445, and GSE109169 datasets by using GEO2R and Graphpad. All these three datasets revealed the up-regulated expression level of NUP37 in patients with BRCA (**Figure 2A**). Further, we turned to the Oncomine database (Richardson Breast 2 Dataset and Curtis Breast Dataset) to mine the expression of NUP37 in BRCA. Consistently with the findings from the GEO database, the expression of NUP37 is upregulated in various subtypes of BRCA when compared with normal breast samples, in two independent studies (**Figures 2B, C**). These results confirmed the overexpression of NUP37 in BRCA. Furthermore, analyses of clinical human tissue specimens indicated that Nup37 protein is also highly expressed in breast cancer patients (**Figure 2D**).

**Figure 2:** The expression level of NUP37 in BRCA *versus* normal samples. **(A)** Expression level of NUP37 in BRCA and normal samples from GEO datasets (GSE73613, GSE109169, GSE41445) (Unpaired t test, Cancer *VS.*. Normal, p*<0.05, p***<0.001). **(B)** Oncomine data mining analysis of NUP37 mRNA levels in Richardson Breast 2 Dataset and **(C)** Curtis Breast Dataset between normal breast *versus* breast cancer subtypes. (Unpaired t test, Cancer *VS*. Normal, p*<0.05, p***<0.001) **(D)** Nup37 protein level in breast cancer tissue *versus* adjacent normal tissue for human tissue microarray staining of 45 patients. The representative image of staining tissue (left) and statistic staining score (right) (Unpaired t test, p***<0.001). Scale bar, 400 μm,above; 100 μm, below.

### High NUP37 Expression Might Be an Indicator of Poor Survival Rate in Patients With Breast Cancer

Subsequently, by use of the Kaplan–Meier plotter online tool, we explored the association between NUP37 expression and the relapse-free survival (RFS) and distant metastasis-free survival (DMFS) in patients with BRCA to evaluate the prognostic value of NUP37. The results showed that high expression of NUP37 was associated with unfavorable RFS (**Figure 3A**), as well as DMFS (**Figure 3B**). Moreover, we generated the corresponding Kaplan-Meier Plotter curves according to the different ER statuses (ER-negative and positive samples) and found that the high expression level of NUP37 was related to the poor prognosis in ER positive samples but not for ER-negative samples (**Figures 3C, D**). Additionally, we applied OncoLnc to assess overall survival (OS) and also observed a similar unfavorable OS trend (**Figure 3E**). Taken together, these data suggested that high expression of NUP37 was significantly associated with a worse survival rate for BRCA patients, which indicated NUP37 might be an indicator of poor prognosis in patients with BRCA.

**Figure 3:** Clinical survival significance of NUP37 expression level in BRCA patients. **(A)** Correlation of NUP37 expression with RFS and **(B)** DMFS using Kaplan–Meier plotter. Statistical significance was estimated using a log-rank test. **(C)** Correlation of NUP37 expression with RFS and **(D)** DMFS curves calculated by Kaplan–Meier plotter for patients with breast cancer classified as ER+ (left) and ER− (right) respectively. Statistical significance was estimated using a log-rank test. **(E)** Kaplan-Meier curve for OS in BRCA patients grouped by the level of NUP37 expression using OncoLnc. Statistical significance was estimated using a log-rank test.

### High NUP37 Expression Might Be Involved in Tumorigenesis by Promoting Cell Growth, Migration, and Stemness

Based on the bioinformatics analysis, we additionally confirmed the expression level of NUP37 in various BRCA cell lines. We found NUP37 to be highly expressed in BRCA cells when compared with MCF10A cells (**Figure 4A**). Next, in order to confirm the functional effects of NUP37 on breast cancer cells, two siRNAs were applied to knockdown of NUP37 in BT-549 and ZR-75-30 cells, which are the top two cell lines with high expression levels of NUP37 in western blot assays (**Figure 4B**). Significantly, cell growth was inhibited following NUP37 knockdown (**Figure 4C**). Also, after NUP37 was downregulated, we observed cell migration was slow down *via* wound-healing assays (**Figure 5A**) and transwell migration assays (**Figure 5B**). Epithelial cell marker occludin, a tight junction protein, is up-regulated, which leads to the gain of cell-cell adhesion, while mesenchymal marker vimentin is decreased (**Figure 5C**). Moreover, expression of the cancer stem cell surface marker CD44^+^CD24^-/low^ subpopulation, which is measured by flow cytometry and mammosphere forming efficiency, was also reduced after NUP37 downregulated (**Figures 5D, E**). The siNUP37 exerts its inhibitory effects on the cell proliferation, migration, EMT, and cell stemness of breast cancer cells, which indicated the oncogenic role of NUP37 in the biological characteristic of breast cancer cells.

**Figure 4:** NUP37 knockdown inhibits BRCA cell growth. **(A)** Western blot analysis confirmed a strong expression of NUP37 protein in the BRCA cells MDA-MB-231, MCF7, BT-549, ZR-75-30, and T47D compared with MCF10A. GAPDH was used as a loading control. **(B)** Western blot analysis of NUP37 protein levels in BT-549 and ZR-75-30 cells transfected with siNUP37 or siRNA control for 72 h. GAPDH was used as a loading control. **(C)** The proliferation of BT-549 and ZR-75-30 cells transfected with siNUP37 or siRNA control for the indicated time was assessed by counting the number of cells. The experiments were performed at least in triplicate, and the results are presented as the mean ± s.d. The data were analyzed by Student’s t-test (**p < 0.01; ***p < 0.001).

**Figure 5:** NUP37 knockdown attenuates BRCA cell migration. **(A)** Scratch assays of BT-549 and ZR-75-30 cells transfected with siNUP37 or siRNA control for 36h and 24h, respectively. Images and Statistical data are shown. Scale bar, 300 μm. **(B)** Transwell assays of BT-549 and ZR-75-30 cells transfected with siNUP37 or siRNA control for 36h and 24h, respectively. Representative images are shown, and the migrated cells were counted. Scale bar, 200 μm. **(C)** Western blot analysis of EMT marker protein levels in BT-549 and ZR-75-30 cells transfected with siNUP37 or siRNA control for 72 h. GAPDH was used as a loading control. **(D)** After transfected with siNUP37 or siRNA control for 72 h, flow cytometry analysis of BT-549 and ZR-75-30 cells stained with antibodies against CD44 and CD24 was performed. **(E)** Mammosphere assay of BT-549 and ZR-75-30 cells transfected with siNUP37 or siRNA control for 7 days. Representative images are shown, and the spheroids were counted. Scale bar, 300 μm. The experiments were performed at least in triplicate, and the results are presented as the mean ± s.d. The data were analyzed by Student’s t-test (*p < 0.05; **p < 0.01; ***p < 0.001).

### Analysis of NUP37 Associated Cellular Molecule and Pathway

To further explore the possible molecule mechanism and signal pathway that cooperates with NUP37 in the regulation of the BRCA process, we used STRING to construct the PPI network. The proteins directly interacted with NUP37, with a high degree in the PPI network including NUP98, NUP160, SEH1L, NUP85, TPR, SEC13, NUP43, NUP133, NUP153, and NUP107 (**Figure 6A**). By way of the Multi Experiment Matrix (MEM), a web tool for mining gene-gene interaction to exhibit co-expressed genes, we found the co-expression genes of NUP37 (**Table 3**). In addition, we performed Metascape analysis found the NUP37 related terms are mainly involved in chaperonin containing TCP1 complex, synthesis of DNA, mismatch repair, mitochondrial translation initiation, NEP/NS2 interacts with the cellular export machinery, exonucleolytic nuclear-transcribed mRNA catabolic process involved in deadenylation-dependent decay, urine ribonucleoside monophosphate metabolic process, DNA replication-independent nucleosome assembly, methylation, cell division, and responses to nutrients (**Figure 6B**). Importantly, we analyzed the top co-expressed genes from **Table 3** by using Xena based on the TCGA-BRCA database, and then we found the expression of PSMG1 is also highly related with NUP37 in BRCA samples with Pearson’s rho 0.8805 and Spearman’s rank rho ρ = 0.4337 (**Figures 6C, D**), and a high expression level of PSMG1 was related to the poor prognosis in ER-positive samples (**Figure 6E**). Taken together, these results indicated PSMG1 might be a molecule that cooperates with NUP37 in the oncogenetic pathway of BRCA.

**Figure 6:** Prediction of potential molecule mechanism of NUP37 in BRCA. **(A)** The proteins directly interacted with NUP37. **(B)** The enrichment and annotation of NUP37-related terms using Metascape analysis. **(C)** Heatmap of the co-expressed relationship between PSMG1 and NUP37 based on TCGA-BRCA database. **(D)** Co-expression analysis of PSMG1 and NUP37. **(E)** Correlation of PSMG1 expression with RFS (left) and DMFS (right) curves calculated by Kaplan–Meier plotter for patients with breast cancer classified as ER+. Statistical significance was estimated using a log-rank test.

**Table 3:** Co-expression genes of NUP37(Top 10).

Score	Gene name	Gene description	Probeset ID
4.95E-76	WDR61	WD repeat domain 61	221532_s_at
7.25E-75	SSBP1	single stranded DNA binding protein 1	202591_s_at
2.83E-73	ATP5F1	ATP synthase, H+ transporting, mitochondrial Fo complex subunit B1	211755_s_at
1.03E-70	PSMG1	proteasome assembly chaperone 1	203405_at
3.02E-70	MRPS23	mitochondrial ribosomal protein S23	223156_at
3.79E-70	ADSL	adenylosuccinate lyase	210250_x_at
1.32E-69	CCT4	chaperonin containing TCP1 subunit 4	200877_at
9.91E-68	MRPL13	mitochondrial ribosomal protein L13	218049_s_at
1.80E-67	CSE1L	chromosome segregation 1 like	201112_s_at
1.76E-66	METTL5	methyltransferase like 5	221570_s_at

## Discussion

Bioinformatics analysis of public data is a useful, effective, and credible approach in cancer research. It is likely to screen possible target molecules of mammary tumorigenesis and identify targets for cancer prevention and treatment.

Actually, by using STRING and Cytoscape to construct the PPI network of DEGs, we got the top 10 core genes located in the key nodes with the highest degrees. Meanwhile, the GO analysis showed that the 138 upregulated DEGs were primarily enriched in the cellular component of the nuclear part and in the biological process of the cell cycle. Then, we did some literature work on these top core genes one by one from highest to lowest degrees. We found that Cdc20 (Cell division cycle protein 20), Cdc42 (Cell division cycle protein 42), NUP37, ANAPC11 (Anaphase-promoting complex subunit 11), TUBA1A (alpha-tubulin), and CENPO (Centromere protein O) have been wildly reported as cell-cycle-related proteins. Among them, Cdc20 (25, 26), Cdc42 (27), and CENPO (28) have been identified as prognostic and predictive biomarkers and therapeutic targets in breast cancer. Thus, we focused on the relatively high degree gene NUP37 to perform further exploration, and we found interesting results in our manuscript. Of note, this does not exclude the possibility that other genes including UBB (Ubiquitin B), PSMC6 (Proteasome 26S subunit, ATPase 6), PEN1 (Penetration 1), HIST1H2BB (Histone Cluster 1 H2B Family Member B) would also play a role in the development of breast cancer. They need to be further explored.

Nuclear pore complexes (NPCs) are supermolecular structures that act as bidirectional nuclear transport channels embedded in the nuclear envelope in eukaryotic cells. NPCs have a diameter of ~0.13 μm and are constructed by the repetition of 32 different proteins termed nucleoporins (Nups) (29). Previously, researchers believed that the primary role of NPCs was to regulate molecular exchange and genetic information transport between the nucleus and cytoplasm (30). Over the last two decades, with increasing understanding of the main geometrical and structural features of NPCs (29, 31), some additional biological functions of certain NPCs have emerged, such as genome organization, the maintenance of genome integrity, and modulation of gene expression by transcriptional regulation related to cell division, cell motility, cell remodeling, and cell differentiation, and this is also linked to several human neoplastic and non-neoplastic diseases (32, 33).

The role of NUP37 has rarely been reported in cancer cells and has never been studied in BRCA previously. In this study, the PPI network showed the top 10 interactions between NUP37 and NUP98, NUP160, SEH1L, NUP85, TPR, SEC13, NUP43, NUP133, NUP153, and NUP107. In solid and hematological tumors, deregulated NUPs, including NUP210, NUP133, NUP107, SEC13, NUP188, NUP93, NUP62, NUP153, TPR, RANBP2, NUP214, NUP98, NUPL2, and RAE1, have been revealed (34, 35). Nup98 (98-kD Nup) is an NPC component that, in addition to its role in nuclear transport, was identified as a transcriptional regulator at gene promoters to control transcription of its target genes in human cells (36). NUP98 is fused to various partner genes in multiple hematopoietic malignancies (37, 38) and colocalizes with the Nup107-160 complex and promotes the cell division process (39). Another nucleoporin, Nup153, is required to recruit the Nup107-160 complex to the inner nuclear membrane for interphasic NPC assembly (40). Nup153 maintains nuclear envelope architecture and is required for cell migration in tumor cells (41). One study demonstrated that NUP160–SLC43A3 is a novel recurrent fusion oncogene in angiosarcoma (42). Nup88 (88-kD Nup) has been found to be overexpressed in numerous malignant neoplasms, indicating that Nup88 may be a potential molecular marker of many malignancies and premalignant dysplasia (43). These findings enhanced the prediction of the regulatory role of NUP37 in the progression of BRCA carcinogenesis. Since we only evaluated NUP37 as a biomarker in BRCA by publicly available database and confirmed the function of NUP37 *in vitro* experiments using breast cancer cell lines, an *in vivo* study and an outcome for breast cancer patients and NUP37 in a prospective data set are further required.

The 26S proteasome is a multisubunit complex composed of the 19S regulatory particles and the core catalytic 20S proteasome, which is responsible for protein degradation. As proteasome assembly chaperone, the PSMG1 binds to the PSMA proteasome subunits, promotes maturation and stability of the 20S proteasome alpha subunits (44). The role of PSMG1 in cancer has barely been reported. One study reported that the amino acid sequence of PSMG1 protein has a potential homology to proteins involved in the cell cycle, and the function of the PSMG1 protein could be related to cell proliferation (45). Moreover, Zhang et al. demonstrated that high expression of POMP (proteasome maturation protein), another proteasome assembly chaperone for 20S proteasome, is involved in the regulation of cell proliferation and significantly correlated with poor relapse-free survival for ER-positive breast cancer patients (46). Otherwise, it is well accepted that the proteasome pathway plays a significant role in oncogenesis by degradation of most tumor suppressors proteins required for cell-cycle progression and mitosis (47). This proteasome-mediated degradation depends on proteasome abundance through the coordinated expression of proteasome subunits and assembly chaperones (48). These evidence suggests that upregulation of PSMG1 may be able to promote tumor growth by activating 20S proteasome assembly and thereby degrading the tumor suppressors. In addition, increasing evidence indicates that mature proteasomes are targeted to the nuclear periphery or transported into the nucleus through the mature nuclear pore complexes (NPCs) (49, 50). Basing on the database, we found that PSMG1 is highly co-expressed with NUP37 in breast cancer and also associated with poor prognosis in ER-positive patients. Thus, we speculated that PSMG1 might be a molecule that cooperates with NUP37 in the oncogenetic pathway of BRCA. As this hypothesis is a novel finding in breast cancer, it is potentially expanding the cellular functions of NUP37 and PSMG1. However, the conclusions in our present study are based on analyses from public data of patient samples, which have limitations. Therefore, to make a stronger elucidation of the connected function of NUP37 and PSMG1 in breast cancer, future exploration would be needed.

Because at least 70% of breast cancers are ERα positive (ERα+) with enhanced ERα expression and ERα signaling, the ERα level is important for the diagnosis and endocrine therapy of BRCA. The NPC transport system plays a critical role in the regulation of the localization of ERα and ERα signaling pathways by the dynamic shuttling of ERα between the cytoplasm and nucleus through recognition of the specific amino acid sequences of NLSs and NESs (51). Our study evaluated the role of NUP37 in BRCA and investigated its potential application as a marker for the preliminary diagnosis and therapy in BRCA. In addition, we found that NUP37 may play a role in the prognosis of BRCA only in ER-positive patients, which indicates that ER signaling may be an underlying target of NUP37. More experimental evidence is needed to verify whether Nup37 mediates the ERα nuclear-cytoplasmic trafficking mechanism in tumorigenesis and the endocrine therapy of BRCA. ERα protein levels and locations, expression of ERα target genes, and estrogen response signal activity require evaluation after NUP37 depletion.

## Data Availability Statement

The raw data supporting the conclusions of this article will be made available by the authors, without undue reservation.

## Author Contributions

KL performed all the bioinformatics analysis. TL did the experimental assays, wrote the manuscript, and supervised the project. All authors contributed to the article and approved the submitted version.

## Funding

This study was supported by the National Natural Science Foundation of China (81903101), Project of Wuhan Municipal Health Commission (WZ18Q02).

## Conflict of Interest

The authors declare that the research was conducted in the absence of any commercial or financial relationships that could be construed as a potential conflict of interest.

## Publisher’s Note

All claims expressed in this article are solely those of the authors and do not necessarily represent those of their affiliated organizations, or those of the publisher, the editors and the reviewers. Any product that may be evaluated in this article, or claim that may be made by its manufacturer, is not guaranteed or endorsed by the publisher.

## References

[1] SiegelRLMillerKDJemalA. Cancer Statistics, 2018. CA Cancer J Clin (2018) 68:7–30. 10.3322/caac.21442 29313949

[2] DonepudiMSKondapalliKAmosSJP. Breast Cancer Statistics and Markers. J Cancer Res Ther (2014) 10:506–11. 10.4103/0973-1482.137927 25313729

[3] DaiYTangYHeFZhangYChengAGanR. Screening and Functional Analysis of Differentially Expressed Genes in EBV-Transformed Lymphoblasts. Virol J (2012) 9:77. 10.1186/1743-422X-9-77 22458412PMC3433351

[4] ZhangCPengLZhangYLiuZLiWChenS. The Identification of Key Genes and Pathways in Hepatocellular Carcinoma by Bioinformatics Analysis of High-Throughput Data. Med Oncol (2017) 34:101. 10.1007/s12032-017-0963-9 28432618PMC5400790

[5] HeRQWuPRXiangXLYangXLiangHWQiuXH. Downregulated miR-23b-3p Expression Acts as a Predictor of Hepatocellular Carcinoma Progression: A Study Based on Public Data and RT-qPCR Verification. Int J Mol Med (2018) 41:2813–31. 10.3892/ijmm.2018.3513 PMC584665429484429

[6] LongJZhangZLiuZXuYGeC. Identification of Genes and Pathways Associated With Pancreatic Ductal Adenocarcinoma by Bioinformatics Analyses. Oncol Lett (2016) 11:1391–7. 10.3892/ol.2015.4042 PMC473432126893748

[7] MaXShangFZhuWLinQ. CXCR4 Expression Varies Significantly Among Different Subtypes of Glioblastoma Multiforme (GBM) and its Low Expression or Hypermethylation Might Predict Favorable Overall Survival. Expert Rev Neurother (2017) 17:941–6. 10.1080/14737175.2017.1351299 28685624

[8] MaQWuXWuJLiangZLiuT. SERP1 is a Novel Marker of Poor Prognosis in Pancreatic Ductal Adenocarcinoma Patients via Anti-Apoptosis and Regulating SRPRB/NF-kappaB Axis. Int J Oncol (2017) 51:1104–14. 10.3892/ijo.2017.4111 PMC559285928902358

[9] PiaoJSunJYangYJinTChenLLinZ. Target Gene Screening and Evaluation of Prognostic Values in non-Small Cell Lung Cancers by Bioinformatics Analysis. Gene (2018) 647:306–11. 10.1016/j.gene.2018.01.003 29305979

[10] DuFLiYZhangWKaleSPMcFerrinHDavenportI. Highly and Moderately Aggressive Mouse Ovarian Cancer Cell Lines Exhibit Differential Gene Expression. Tumour Biol (2016) 37:11147–62. 10.1007/s13277-015-4518-4 PMC529213326935058

[11] MenCDLiuQNRenQ. A Prognostic 11 Genes Expression Model for Ovarian Cancer. J Cell Biochem (2018) 119:1971–8. 10.1002/jcb.26358 28817186

[12] HampoelzBAndres-PonsAKastritisPBeckM. Structure and Assembly of the Nuclear Pore Complex. Annu Rev Biophys (2019) 48:515–36. 10.1146/annurev-biophys-052118-115308 30943044

[13] RaicesMD'AngeloMA. Nuclear Pore Complexes and Regulation of Gene Expression. Curr Opin Cell Biol (2017) 46:26–32. 10.1016/j.ceb.2016.12.006 28088069PMC5505778

[14] ChakrabortyPWangYWeiJHvan DeursenJYuHMalureanuL. Nucleoporin Levels Regulate Cell Cycle Progression and Phase-Specific Gene Expression. Dev Cell (2008) 15:657–67. 10.1016/j.devcel.2008.08.020 PMC283557519000832

[15] TamuraKFukaoYIwamotoMHaraguchiTHara-NishimuraI. Identification and Characterization of Nuclear Pore Complex Components in Arabidopsis Thaliana. Plant Cell (2010) 22:4084–97. 10.1105/tpc.110.079947 PMC302718321189294

[16] BilokapicSSchwartzTU. Molecular Basis for Nup37 and ELY5/ELYS Recruitment to the Nuclear Pore Complex. Proc Natl Acad Sci USA (2012) 109:15241–6. 10.1073/pnas.1205151109 PMC345832122955883

[17] LoiodiceIAlvesARabutGVan OverbeekMEllenbergJSibaritaJB. The Entire Nup107-160 Complex, Including Three New Members, is Targeted as One Entity to Kinetochores in Mitosis. Mol Biol Cell (2004) 15:3333–44. 10.1091/mbc.e03-12-0878 PMC45258715146057

[18] LuoXLiuYFengWLeiLDuYWuJ. NUP37, a Positive Regulator of YAP/TEAD Signaling, Promotes the Progression of Hepatocellular Carcinoma. Oncotarget (2017) 8:98004–13. 10.18632/oncotarget.20336 PMC571670929228669

[19] ChenJWoDaMaEnYanHPengJZhuW. Deletion of Low-Density Lipoprotein-Related Receptor 5 Inhibits Liver Cancer Cell Proliferation via Destabilizing Nucleoporin 37. Cell Comm Signal (2019) 17:174. 10.1186/s12964-019-0495-3 PMC693519931881970

[20] HuangLWangTWangFHuXZhanGJinX. NUP37 Silencing Induces Inhibition of Cell Proliferation, G1 Phase Cell Cycle Arrest and Apoptosis in non-Small Cell Lung Cancer Cells. Pathol Res Pract (2020) 216:152836. 10.1016/j.prp.2020.152836 32014308

[21] HiranoYHendilKBYashirodaHIemuraSNaganeRHiokiY. A Heterodimeric Complex That Promotes the Assembly of Mammalian 20S Proteasomes. Nature (2005) 437:1381–5. 10.1038/nature04106 16251969

[22] WuYSarkissyanMVadgamaJV. Epithelial-Mesenchymal Transition and Breast Cancer. J Clin Med (2016) 5:13. 10.3390/jcm5020013 PMC477376926821054

[23] ThieryJPAcloqueHHuangRYNietoMA. Epithelial-Mesenchymal Transitions in Development and Disease. Cell (2009) 139:871–90. 10.1016/j.cell.2009.11.007 19945376

[24] ButtiRGunasekaranVPKumarTVSBanerjeePKunduGC. Breast Cancer Stem Cells: Biology and Therapeutic Implications. Int J Biochem Cell Biol (2019) 107:38–52. 10.1016/j.biocel.2018.12.001 30529656

[25] AlfarsiLHAnsariRECrazeMLTossMSMasisiBEllisIO. CDC20 Expression in Oestrogen Receptor Positive Breast Cancer Predicts Poor Prognosis and Lack of Response to Endocrine Therapy. Breast Cancer Res Treat (2019) 178:535–44. 10.1007/s10549-019-05420-8 31471836

[26] ChengLHuangYZChenWXShiLLiZZhangX. Cell Division Cycle Proteinising Prognostic Biomarker of Breast Cancer. Biosci Rep (2020) 40:BSR20191227. 10.1042/BSR20191227 32285914PMC7201563

[27] ZhangYLiJLaiXNJiaoXQXiongJPXiongLX. Focus on Cdc42 in Breast Cancer: New Insights, Target Therapy Development and Non-Coding RNAs. Cells (2019) 8:146. 10.3390/cells8020146 PMC640658930754684

[28] ZhangSXieYTianTYangQZhouYQiuJ. High Expression Levels of Centromere Protein A Plus Upregulation of the Phosphatidylinositol 3-Kinase/Akt/mammalian Target of Rapamycin Signaling Pathway Affect Chemotherapy Response and Prognosis in Patients With Breast Cancer. Oncol Lett (2021) 21:410. 10.3892/ol.2021.12671 33841571PMC8020387

[29] HoelzAGlavyJSBeckM. Toward the Atomic Structure of the Nuclear Pore Complex: When Top Down Meets Bottom Up. Nat Struct Mol Biol (2016) 23:624–30. 10.1038/nsmb.3244 PMC515657327273515

[30] OnischenkoEWeisK. Nuclear Pore Complex-a Coat Specifically Tailored for the Nuclear Envelope. Curr Opin Cell Biol (2011) 23:293–301. 10.1016/j.ceb.2011.01.002 21296566PMC3109177

[31] MaJKelichJMJunodSLYangW. Super-Resolution Mapping of Scaffold Nucleoporins in the Nuclear Pore Complex. J Cell Sci (2017) 130:1299–306. 10.1242/jcs.193912 PMC539977928202688

[32] D'AngeloMA. Nuclear Pore Complexes as Hubs for Gene Regulation. Nucleus (2018) 9:142–8. 10.1080/19491034.2017.1395542 PMC597325929095096

[33] NofriniVDi GiacomoDMecucciC. Nucleoporin Genes in Human Diseases. Eur J Hum Genet (2016) 24:1388–95. 10.1038/ejhg.2016.25 PMC502767627071718

[34] ItohGSuginoSIkedaMMizuguchiMKannoSAminMA. Nucleoporin Nup188 is Required for Chromosome Alignment in Mitosis. Cancer Sci (2013) 104:871–9. 10.1111/cas.12159 PMC765713323551833

[35] HaoQZhangQLiCWeiSLiQSongY. A Novel Variant Translocation (1;9)(P22;Q34) Resulting in a DEK/NUP214 Fusion Gene in a Patient With Acute Myeloid Leukemia: A Case Report. Oncol Lett (2017) 14:7021–4. 10.3892/ol.2017.7133 PMC575488329344131

[36] FranksTMBennerCNarvaizaIMarchettoMCYoungJMMalikHS. Evolution of a Transcriptional Regulator From a Transmembrane Nucleoporin. Genes Dev (2016) 30:1155–71. 10.1101/gad.280941.116 PMC488883727198230

[37] XuHValerioDGEisoldMESinhaAKocheRPHuW. NUP98 Fusion Proteins Interact With the NSL and MLL1 Complexes to Drive Leukemogenesis. Cancer Cell (2016) 30:863–78. 10.1016/j.ccell.2016.10.019 PMC550128227889185

[38] FranksTMMcCloskeyAShokirevMNBennerCRathoreAHetzerMW. Nup98 Recruits the Wdr82-Set1A/COMPASS Complex to Promoters to Regulate H3K4 Trimethylation in Hematopoietic Progenitor Cells. Genes Dev (2017) 31:2222–34. 10.1101/gad.306753.117 PMC576976729269482

[39] Morchoisne-BolhySGeoffroyMCBouhlelIBAlvesAAudugeNBaudinX. Intranuclear Dynamics of the Nup107-160 Complex. Mol Biol Cell (2015) 26:2343–56. 10.1091/mbc.E15-02-0060 PMC446295025904327

[40] VollmerBLorenzMMoreno-AndresDBodenhoferMDe MagistrisPAstrinidisSA. Nup153 Recruits the Nup107-160 Complex to the Inner Nuclear Membrane for Interphasic Nuclear Pore Complex Assembly. Dev Cell (2015) 33:717–28. 10.1016/j.devcel.2015.04.027 26051542

[41] ZhouLPanteN. The Nucleoporin Nup153 Maintains Nuclear Envelope Architecture and is Required for Cell Migration in Tumor Cells. FEBS Lett (2010) 584:3013–20. 10.1016/j.febslet.2010.05.038 20561986

[42] ShimozonoNJinninMMasuzawaMMasuzawaMWangZHiranoA. NUP160-SLC43A3 is a Novel Recurrent Fusion Oncogene in Angiosarcoma. Cancer Res (2015) 75:4458–65. 10.1158/0008-5472.CAN-15-0418 26527604

[43] HashizumeCNakanoHYoshidaKWongRW. Characterization of the Role of the Tumor Marker Nup88 in Mitosis. Mol Cancer (2010) 9:119. 10.1186/1476-4598-9-119 20497554PMC2890605

[44] HiranoYHayashiHIemuraSHendilKBNiwaSKishimotoT. Cooperation of Multiple Chaperones Required for the Assembly of Mammalian 20S Proteasomes. Mol Cell (2006) 24:977–84. 10.1016/j.molcel.2006.11.015 17189198

[45] Vidal-TaboadaJMLuAPiqueMPonsGGilJOlivaR. Down Syndrome Critical Region Gene 2: Expression During Mouse Development and in Human Cell Lines Indicates a Function Related to Cell Proliferation. Biochem Biophys Res Commun (2000) 272:156–63. 10.1006/bbrc.2000.2726 10872820

[46] ZhangXSchulzREdmundsSKrugerEMarkertEGaedckeJ. MicroRNA-101 Suppresses Tumor Cell Proliferation by Acting as an Endogenous Proteasome Inhibitor via Targeting the Proteasome Assembly Factor POMP. Mol Cell (2015) 59:243–57. 10.1016/j.molcel.2015.05.036 26145175

[47] NaujokatCHoffmannS. Role and Function of the 26S Proteasome in Proliferation and Apoptosis. Lab Invest (2002) 82:965–80. 10.1097/01.LAB.0000022226.23741.37 12177235

[48] RousseauABertolottiA. Regulation of Proteasome Assembly and Activity in Health and Disease. Nat Rev Mol Cell Biol (2018) 19:697–712. 10.1038/s41580-018-0040-z 30065390

[49] WendlerPEnenkelC. Nuclear Transport of Yeast Proteasomes. Front Mol Biosci (2019) 6:34. 10.3389/fmolb.2019.00034 31157235PMC6532418

[50] SavulescuAFShorerHKleifeldOCohenIGruberRGlickmanMH. Nuclear Import of an Intact Preassembled Proteasome Particle. Mol Biol Cell (2011) 22:880–91. 10.1091/mbc.e10-07-0595 PMC305771121289101

[51] Tecalco-CruzACPerez-AlvaradoIARamirez-JarquinJORocha-ZavaletaL. Nucleo-Cytoplasmic Transport of Estrogen Receptor Alpha in Breast Cancer Cells. Cell Signal (2017) 34:121–32. 10.1016/j.cellsig.2017.03.011 28341599

